# Cr–Diamond/Cu Composites with High Thermal Conductivity Fabricated by Vacuum Hot Pressing

This article has been retracted.

**DOI:** 10.3390/ma17153711

**Published:** 2024-07-26

**Authors:** Qiang Xu, Xiaodie Cao, Yibo Liu, Yanjun Xu, Jiajun Wu

**Affiliations:** 1 Central Iron & Research Institute, Beijing 100081, China; xuqiang@gangyan-diamond.com (Q.X.); liuyibo@gangyan-diamond.com (Y.L.); 2 Beijing Gang Yan Diamond Products Company, Beijing 102200, China; 3 College of Engineering, Shantou University, Shantou 515063, China; 23xdcao@stu.edu.cn

**Keywords:** Cr–diamond/Cu, interface structure, thermal conductivity, thermal expansion coefficient, fracture mechanism

## Abstract

Chromium-plated diamond/copper composite materials, with Cr layer thicknesses of 150 nm and 200 nm, were synthesized using a vacuum hot-press sintering process. Comparative analysis revealed that the thermal conductivity of the composite material with a Cr layer thickness of 150 nm increased by 266%, while that with a Cr layer thickness of 200 nm increased by 242%, relative to the diamond/copper composite materials without Cr plating. This indicates that the introduction of the Cr layer significantly enhanced the thermal conductivity of the composite material. The thermal properties of the composite material initially increased and subsequently decreased with rising sintering temperature. At a sintering temperature of 1050 °C and a diamond particle size of 210 μm, the thermal conductivity of the chromium-plated diamond/copper composite material reached a maximum value of 593.67 W∙m^−1^∙K^−1^. This high thermal conductivity is attributed to the formation of chromium carbide at the interface. Additionally, the surface of the diamond particles in contact with the carbide layer exhibited a continuous serrated morphology due to the interface reaction. This “pinning effect” at the interface strengthened the bonding between the diamond particles and the copper matrix, thereby enhancing the overall thermal conductivity of the composite material.

## 1. Introduction

With the rapid advancement of microelectronics technology, semiconductor chips and integrated circuits are being utilized to achieve enhanced computing speeds and more intricate functionalities. Core electronic devices at both the chip and module levels continue to evolve towards smaller dimensions, functional integration, and higher power density. Electronic devices are progressively gaining greater potency in various high-tech sectors such as national defense, the electronics industry, new energy, aerospace, etc., with an increasing level of integration. Consequently, heat dissipation has emerged as a pivotal concern that hampers the progress of these industries [1]. Hence, in the design of high-performance electronic packaging, there is an escalating demand for core chip heat-dissipation materials that possess stringent requirements pertaining to thermal conductivity (TC), density, and thermal expansion coefficients [2].

Diamond is a naturally occurring substance known for its exceptional hardness and high thermal conductivity, ranging from 1200 W∙m^−1^∙K^−1^ to 2000 W∙m^−1^∙K^−1^. It also exhibits a low thermal expansion coefficient of 1 × 10^−6^K^−1^ and a relatively small density of 3.52 g∙cm^−3^ [3]. With advancements in artificial synthesis technology, the price of diamond particles has gradually decreased, making the substance even more cost-effective compared to high-purity tungsten powder. Therefore, diamond-reinforced metal matrices (such as Al, Cu, and Ag) have the potential to produce composites with excellent thermal conductivity, low expansion properties, and competitive pricing [4]. Among these matrix materials, copper stands out due to having the second-highest thermal conductivity after silver among non-noble metals, and its relatively low thermal expansion coefficient when compared to aluminum [5]. Consequently, diamond/copper composite materials are considered promising candidates for next-generation electronic packaging heat-dissipation materials, and have garnered significant attention in recent years. Currently, reported values for the thermal conductivity of diamond/copper composites range from 400 W∙m^−1^∙K^−1^ to 930 W∙m^−1^∙K^−1^ [6,7,8,9]. Wang et al. [10] showed that, at maximum diamond grain size (246 um), the interfacial thermal conductivity of these composite materials is about 4 MW∙m^−2^∙K^−1^, and thermal conductivity is around 400 W/m.K. Ideal Cu–diamond composites have zero interfacial heat, and have calculated thermal conductivity values as high as 840.9 W∙m^−1^∙K^−1^. In the presence of a TiC transition layer, the interfacial thermal conductivity decreases with the increase in the thickness of the transition layer, and the calculated value of the thermal conductivity of the composite material is the highest at the transition layer thickness of 10 nm, reaching 747.6 W∙m^−1^∙K^−1^.

The preparation processes of diamond/copper composites are diverse, encompassing various methods such as spark plasma sintering, high-temperature and high-pressure techniques, metal infiltration, vacuum hot-pressed sintering, etc. Recent research reports have also mentioned alternative methods, including hot forging [5,8], electrodeposition [9,11], ultrasonic consolidation [10], and laser printing [11,12], among others. Hot-pressed sintering (HP), a powder metallurgy process capable of maintaining simultaneous pressure and temperature conditions, finds extensive applications in the fabrication of metal matrix composites. Its advantages lie in the simplicity of the required equipment and the flexibility of the preparation process, which enables achieving phase combination at temperatures below the melting point of low-melting-point phases within composite materials. A variation of this approach is vacuum hot-pressed sintering (VHP), which involves performing hot-pressed sintering under a vacuum atmosphere.

Compared to the spark plasma sintering (SPS) method, the VHP method requires a longer sintering time to allow sufficient time for interface diffusion or chemical reactions to occur. However, in the case of diamond/copper composites, the main reason for poor interface bonding is the lack of chemical reaction and wetting adhesion between the diamond and copper. Simply increasing the sintering time has a limited impact on improving interface contact. Schubert et al. [13] sintered a 42 vol.% diamond/copper–chromium composite at 950 °C and extended the sintering time from 20 min to 30 min. This resulted in an increase in thermal conductivity from 590 W m^−1^∙K^−1^ to 639 W∙m^−1^∙K^−1^, representing an improvement of 8.3%. Currently, the thermal conductivity of diamond/copper composites can reach up to 1000 W∙m^−1^∙K^−1^, with values exceeding 700 W m^−1^∙K^−1^ mainly achieved through the gas pressure infiltration (GPI) method [14]. In comparison with the GPI method, VHP offers more precise control over the quality and density of the diamond particles and the copper matrix in composite materials without requiring prefabricated billets, while also being cost-effective due to cheaper equipment costs. Therefore, utilizing the VHP method for preparing diamond/copper composites holds promising prospects for applications in the consumer electronics market, considering both performance and price.

To enhance the wettability between diamond particles and the matrix, interface modification treatments are required for diamond/copper composites [1]. Various methods of metal coating are commonly employed on diamond surfaces, including chemical plating, salt-bath plating, vacuum micro-evaporation coating, magnetron sputtering, and diffusion techniques. In comparison to copper matrix alloying, the metallization of the diamond surface can further improve the thermal conductivity of the composite; the method allows us to adjust the composition and proportion of the interface phase through variations in coating temperature and duration. Metal carbide-forming elements, such as Ti [15], Zr [16], Cr [17], Mo [18], W [19], etc., are typically chosen based on considerations of phonon velocity, thermal conductivity, and solubility in the matrix. Ren et al. [20] compared the effects of Cr coating and Ti coating modifications under identical conditions and observed that Cr coating effectively reduces interfacial thermal resistance to a greater extent. Chromium-coated diamond/Cu composites exhibit a thermal conductivity (528 W∙m^−1^∙K^−1^) that is 51% higher than that achieved with diamond (Ti)/Cu composites and three times higher than those without any interface modification. Additionally, another method to enhance bonding between diamond particles and the matrix is by varying the load during the sintering process. This approach is inspired by diffusion bonding techniques, which have shown that adjusting the load can significantly improve the bonding quality by influencing the diffusion and interaction at the interface [21]. The application of varying loads during the vacuum hot-press process could potentially lead to better interface contact and bonding strength, thereby further enhancing the thermal conductivity and mechanical properties of diamond/copper composites.

Liu et al. [22] found that the partial transformation of Cr coating to Cr_3_C_2_ is beneficial to the heat exchange between diamond and copper. The thermal conductivity of chromium-coated diamond/Cu composites prepared by Chu et al. [23] with Cr_3_C_2_ in the interface layer was 284 W∙m^−1^∙K^−1^. The thermal characteristics of Cr-modified diamond/Cu composites are highly dependent on the microstructural attributes of the interface layer. The composite prepared by Kang et al. [24] with a thermal conductivity of 562 W∙m^−1^∙K^−1^ mainly contained Cr_3_C_7_ as the carbide at the interface. Coatings of elements such as W and Ti can even form a multi-phase interface of multiple carbides with higher thermal conductivity.

The vacuum hot-press sintering process for the preparation of tool-grade Cr–diamond/Cu composites has simple equipment requirements, low production costs, and good mechanical properties [25]. It has been maturely applied to tools such as drills and saw blades. However, the diamond volume fraction in such materials generally does not exceed 20%, and it is difficult to reach a thermal conductivity of 400 W∙m^−1^∙K^−1^ [26]. There is a lack of systematic and feasible process designs for preparing high-volume-fraction, high-thermal-conductivity diamond/copper composites using hot-press sintering. This study prepared diamond/Cu composites with different particle sizes and different thicknesses of chromium coatings and investigated the effects of different process parameters on the microstructure, thermal conductivity, and mechanical properties of these composites.

## 2. Materials and Methods

### 2.1. Preparation of Cr–Diamond/Cu Composites

In this study, MBD6 artificial diamond particles with particle sizes of 325/400 mesh (38 µm~45 μm), 170/200 mesh (75 µm~90 μm), and 70/80 mesh (180 µm~212 μm) were used as reinforcement materials for the composite. The diamond particles used in the experiment were divided into bare diamond particles and diamond particles with a pre-plated Cr layer on the surface of the bare diamond particles. Commercially available electrolytic copper powder (99.9 wt%) was used as the matrix material. The electrolytic copper powder particles have a dendritic shape and a laser particle size of 35 μm. The diamond/copper composite was prepared using a ZM-34-10 vacuum-protected atmosphere sintering furnace produced by Shanghai Chenhua Technology (Shanghai, China). First, certain masses of copper powder and diamond particles were weighed and mixed, and the evenly mixed powder material was loaded into a graphite mold, smoothed, and compacted. The loaded graphite mold was placed on the lifting platform of the vacuum-protected atmosphere sintering furnace, and the pressure system was adjusted to fix the graphite mold in the heating zone of the equipment. Then, the furnace chamber was evacuated, and once the pressure dropped below 101 Pa, the heating program was initiated to heat the sample. Based on previous experimental results and a literature analysis, the sintering temperature range was set to 850 °C~1100 °C, the pressure was set to 20 MPa~30 MPa, and the holding time was 30 min. After the holding time ended, the heating was stopped, and the pressure was maintained for 60 min to reduce the pores formed by interface shrinkage during the cooling process. After the pressure was maintained, the furnace was cooled to room temperature with the sample inside.

### 2.2. Material Characterization

The cross-sections of the diamond particles and the bending fracture morphology of the composite were observed using an FEI Nova nanoSEM450 field-emission scanning electron microscope (SEM) (Hillsboro, OR, USA). The element distribution was determined using an X-Max50 X-ray energy-dispersive spectroscopy (EDS) analyzer (Oxford, Oxfordshire, UK) configured with the scanning electron microscope. The phase compositions of the composites synthesized at different temperatures (850 °C, 950 °C, 1050 °C) were analyzed by X-ray diffraction (XRD). The nitrogen content in the diamond particles was measured using a Leco TC600 nitrogen oxide analyzer (San Jose, CA, USA). The thermal diffusivity α of the composite was measured by the flash method using a NETZSCH LFA457 laser flash apparatus (LFA) (Seer, Germany). The dilation curve of the diamond/copper composite was tested using a NETZSCH DIL 402SU dilatometer (Seer, Germany). A CMT4300 universal electronic testing machine (Shanghai, China) was used to perform a three-point bending test to test the bending performance of the composite.

## 3. Results and Discussion

### 3.1. Properties of Composites Prepared with Different Chromium Layer Thicknesses

Cr–diamond/copper composites with Cr layer thicknesses of 150 nm and 200 nm were prepared by vacuum hot-press sintering at 850 °C and 20 MPa, respectively. The diamond particles used had a particle size of 45 μm and a volume fraction of 60 vol.%. The thermal conductivity of the composites is shown in Table 1. Compared to the thermal conductivity of the diamond/copper composite without Cr plating, the thermal conductivity of the composite with a pre-plated Cr layer thickness of 150 nm increased by 266%, and the thermal conductivity of the composite with a pre-plated Cr layer thickness of 200 nm increased by 242%, indicating that the introduction of the Cr layer effectively improved the thermal conductivity of the composite, aligning with Ukhina’s research findings [27]. Additionally, the material with a sintering temperature of 850 °C and a Cr layer thickness of 150 nm exhibited slightly higher thermal conductivity than the composite with a Cr layer thickness of 200 nm.

### 3.2. Interface Structure of Cr–Diamond/Copper Composite Material

Figure 1 shows the surface morphology of the diamond/copper composite materials, in which the diamond particles maintain their original tetradecahedral shape. As can be seen in Figure 1a, the reinforced diamond particle is mechanically embedded in the matrix, and the diamond surface is very smooth. However, in Figure 1b, the diamond particle surface in the chromium-plated diamond/copper composite is uniformly covered by a carbide layer formed by the reaction between the Cr layer and the diamond surface. The reaction products accumulated on the diamond particle surface, forming a patterned structure, as shown in Figure 2b.

To investigate the interface of the composite material, the cross-section of the fractured diamond particles on the fracture surface of the composite material was observed. As can be seen in Figure 3a, the copper matrix and the reinforced diamond particles are tightly connected, with an interfacial transition layer, no gap, and a flat interface. This indicates a strong metallurgical bond between the diamond particles and the copper matrix, which is crucial for enhancing the thermal conductivity and mechanical strength of the composite. In Figure 3b, irregular particulate reaction products can clearly be observed growing from the diamond particle side in the matrix direction, and the thickest part of the reactant in the interfacial layer does not exceed 1 μm. These reaction products are likely chromium carbides, formed due to the interaction between the chromium coating on the diamond particles and the copper matrix [28]. The presence of these reaction products further reinforces the interface by creating a mechanical interlock, which contributes to the overall stability and performance of the composite material.

Furthermore, the interface modification of the composite material was achieved by chromium plating on the surface of the diamond particles. The composition, thickness, and distribution of the carbides formed at the interface significantly affect the interfacial thermal resistance of the composite. The interfacial structure of chromium-plated diamond/copper composites can exist in various forms, such as diamond–carbide–chromium–copper, diamond–carbide–copper, and diamond–carbide–copper–chromium alloy–copper. The carbides formed from the reaction between the chromium layer and diamond can include Cr_3_C_2_, Cr_7_C_3_, and Cr_23_C_6_. In this study, EDS and XRD analyses were performed on diamond particles extracted from preliminary experimental samples, as shown in Figure 4 and Figure 5. The EDS images reveal a uniform distribution of Cr elements on the surface of the diamond particles, indicating the successful deposition of the chromium coating. From Figure 5, it is evident that Cr_3_C_2_ exhibits distinct diffraction peaks at all temperatures, confirming that Cr_3_C_2_ is the primary carbide phase.

To further investigate the interface structure of the composite material, an EDS micro-interface scan was performed on the composites, and the results are shown in Figure 6. As can be seen from the interface scan result in Figure 6a, the left side is a C element, the right side is a Cu element, and the Cr element layer is evenly and continuously positioned between the diamond particle and the copper matrix, with no sign of Cr diffusion into the matrix.

Upon observation, it was found that the boundary between Cr and Cu contact is undulating. This is analyzed as being due to the granular transition layer formed by Cr at the interface, where differences in the size and shape of the particles result in a serrated boundary at the particle connections. During the preparation of the composite material through vacuum hot pressing, the matrix fills in the depressions and voids at the interface. This filling process not only improves physical contact, but also minimizes the presence of voids, which can act as sites for crack initiation and propagation [29], thereby improving the durability and reliability of the composite material.

Figure 6b shows the line distribution of the interface elements. It can be clearly observed from the figure that the Cr element is uniformly distributed at the interface, and at the same detection site, there is also a strong signal for the C element. This result confirms that the interface layer is a reaction product of Cr and C elements, and the thickness of this interface transition layer is approximately 650 nm. Therefore, based on the calculation of the interface thermal resistance of the composite material [30], the interface thermal resistance of the chromium-plated diamond/copper composite material is $3.94\times 10^{-8}\;m^{2}\cdot K\cdot W^{-1}$ . Calculations using the H-J model and the DEM model yield theoretical thermal conductivities of 797.4 W∙m^−1^∙K^−1^ and 711.7 W∙m^−1^∙K^−1^ for the material, respectively.

### 3.3. Thermal Conductivity and Its Influencing Mechanism in Cr–Diamond/Copper Composite Materials

Table 2 summarizes the test and calculation results of the thermal-conductivity-related parameters of the chromium-plated diamond/copper composite materials prepared under different process parameters. As can be seen from the table, at 850 °C, the thermal conductivity of the chromium-plated diamond/copper composite material is 417 W∙m^−1^∙K^−1^, significantly higher than the thermal conductivity of 127 W∙m^−1^∙K^−1^ for the unplated diamond/copper composite material sample under the same conditions, representing an increase of more than 2 times. This is because the introduction of the chromium layer effectively reduces defects such as interfacial pores, which in turn helps reduce the interfacial [28] thermal resistance and increase the thermal conductivity of the composite material.

When the sintering temperature exceeds 1050 °C, increasing the sintering temperature or changing the sintering pressure does not significantly change the thermal conductivity of the samples. The thermal conductivity value remains stable at approximately 590 W∙m^−1^∙K^−1^, which is 71% and 80% of the theoretical thermal conductivity calculated using the H-J model and the DEM model, respectively. The thermal conductivity of the composite material fails to reach the expected level of the theoretical value. On one hand, as can be seen from Table 2, the samples do not reach a completely dense state, and the existence of internal pores and other defects hinders heat transfer, resulting in a decrease in the thermal conductivity of the material. On the other hand, when establishing the interfacial thermal resistance model for calculating the theoretical thermal conductivity of the composite material, it was assumed that the composition and thickness of the transition layer at the interface were uniform. However, as seen in the interface morphology in Figure 3, the cross-section of the transition layer formed by chromium elements at the interface is serrated, and the actual interface layer is not a uniform lamellar structure. The larger interfacial contact area leads to a higher interfacial thermal resistance, which in turn causes the actual thermal conductivity of the sample to be lower than the theoretical value.

Typically, the operating temperature of electronic components ranges from 25 °C to 300 °C (298 K~573 K) [31], and testing the thermal conductivity within this range is crucial for evaluating the feasibility of diamond/copper composite materials under different environmental temperatures. Table 3 shows the thermal diffusivity of chromium-plated diamond/copper composite materials at temperatures ranging from 298 K to 573 K. The data in the table indicate that the thermal diffusivity of the composite material decreases as the test temperature increases. For composite materials prepared with the same diamond particle sizes, there are significant differences in the rate of decrease in thermal diffusivity as the temperature rises from 298 K to 373 K depending on the preparation process, and the greater the initial thermal diffusivity of the sample, the greater the rate of decrease. As the temperature further increases, the rate of decrease in thermal diffusivity does not vary with the preparation process. As the temperature rises from 373 K to 473 K, the rate of decrease in thermal diffusivity for samples with two different particle sizes is 20% and 24%, respectively. When the temperature increases from 473 K to 573 K, the rates of decrease are 15% and 19%, respectively. In comparison, the thermal diffusivity of the composite material prepared with diamond particles of 210 μm decreases faster with temperature. Over the entire temperature range from 298 K to 573 K, the thermal diffusivity of the chromium-plated diamond 210 μm/copper composite material decreases by 60%.

The thermal conductivity of composite materials is a result of the combined effects of density, thermal diffusivity, and specific heat capacity. Since the density of solid materials is minimally affected by temperature and thermal diffusivity, the impact of density on the thermal conductivity of composite materials can be ignored, and the change in specific heat capacity with temperature needs to be considered. Table 4 shows the specific heat capacity of the composite materials measured by laser flash analysis in the range of 298 K to 573 K. It can be seen from the table that the specific heat capacity of the composite materials increases with the increase in test temperature, and the specific heat capacity at 573 K is about 1.5 to 2 times that at 298 K.

Figure 7 depicts the thermal conductivity of the chromium-plated diamond/copper composite materials within the temperature range of 298 K to 573 K. It can be observed from the figure that the thermal conductivity of the composite materials decreases with the increase in test temperature, but the rate of decline in thermal conductivity varies. As the test temperature increases, the rate of decline in thermal conductivity slows. When the test temperature rises from 298 K to 373 K, the thermal conductivity of the composite materials declines faster. Within this temperature range, the rate of decline in thermal conductivity is similar for composite materials with the same diamond particle size prepared under the same sintering pressure, but different sintering temperatures. However, under the same sintering temperature, the rate of decline in thermal conductivity differs significantly for composite materials prepared under different sintering pressures. This indicates that the sensitivity of the thermal conductivity of chromium-plated diamond/copper composite materials to temperature change is related to their sintering pressure. With higher sintering pressure, the thermal conductivity of the prepared composite materials decreases faster as the ambient temperature increases.

Although the thermal conductivity of the chromium-plated diamond/copper composite materials decreases with the increase in test temperature, their thermal conductivity at 300 °C ranges from 400 W∙m^−1^∙K^−1^ to 500 W∙m^−1^∙K^−1^, which is relatively high compared to that of currently commercially available electronic packaging heat-dissipation materials (generally below 400 W∙m^−1^∙K^−1^). This can satisfy the heat-dissipation requirements of the internal components in most electronic devices during operation (the internal environmental temperature of a device during normal operation is between 50 °C and 300 °C).

### 3.4. Thermal Expansion Coefficient of Cr–Diamond/Copper Composite Materials

Table 5 shows the average thermal expansion coefficients of chromium-plated diamond/copper composite materials in the range of 298 K to 573 K. Figure 8 depicts the thermal expansion performance curve of chromium-plated diamond/copper composite materials prepared by vacuum hot pressing. The thermal expansion coefficient of the composite material increases with the increase in temperature, consistent with the Gruneisen theory. After the temperature reaches 373 K, the growth rate of CTE values decreases. This is because, in the composite material, thermal stress manifests as tensile stress in the copper matrix and compressive stress in the diamond particles of the reinforcement. When the sample is heated to room temperature, the residual stress generated during sample preparation is released, thus promoting the increase in CTE values. At high temperatures, as residual stress reduces, it no longer contributes to the expansion of the sample. Therefore, between 373 K and 573 K, the growth rate of CTE values decreases.

Furthermore, according to the data in Table 5, the average thermal expansion coefficients of the composite materials prepared at the same sintering temperature are similar. As observed in Figure 8, when the test temperature is relatively low, the thermal expansion coefficients of the composite materials prepared at the same sintering temperature show significant differences. However, as the temperature increases, the thermal expansion coefficients of the samples tend to converge.

### 3.5. Fracture Mechanism of Cr–Diamond/Copper Composite Materials

Figure 9, Figure 10 and Figure 11 show the fracture morphologies of samples sintered at 850 °C, 1050 °C, and 1100 °C, respectively. From Figure 8, it can be observed that samples No.1 and No.2 prepared at 850 °C mainly exhibit intergranular fracture. At this temperature, the copper matrix is in the bonding stage, with small grain size and no significant change in particle morphology. In Figure 9b, diamond particles are embedded in the copper matrix, maintaining their original tetradecahedral morphology. The (100) face of the diamond is smooth, and a small amount of matrix is attached to the (111) face. There are voids at the interface between the matrix and diamond particles, and interfacial cracking is the main reason for the intergranular fracture of the composite material [32].

However, in Figure 9d, it can be observed that adhesion is formed between the modified diamond and the copper matrix in sample No. 2, with significantly reduced interfacial voids. Compared to sample No. 1, the interfacial bonding is tighter, indicating that the addition of chromium is beneficial for improving the interfacial bonding state. As the sintering temperature increases, the matrix grains grow, and in addition to the intergranular fracture characteristics of the composite material, as shown in Figure 10, some small dimples appear in the matrix, indicating ductile fracture in the matrix and increased material ductility. A small number of diamond particles are broken, and some diamond particle surfaces retain residual copper matrix, indicating an increase in the interfacial bonding force of the material.

Combining the interface morphology of the composite material shown in Figure 3 and the surface morphology of diamond particles in Figure 12, it can be seen that the added Cr layer reacts with the diamond particle surface to form interfacial carbides. The morphology of the carbides is continuous irregular particles, and the part of the diamond particle surface in contact with the carbide layer also appears as a continuous zigzag shape due to the presence of interfacial reactions. This indicates that the interfacial reaction results in the formation of a “pinning effect” at the interface, strengthening the bonding between the diamond particles and the copper matrix [31]. The improvement in interfacial bonding force leads to an enhancement in the bending performance of the composite material. However, carbides are brittle materials, as shown by the carbide layer on the surface of the diamond particles in Figure 12; after being loaded with external forces, a small amount of the carbide layer fractures and peels off. This may be due to the thick local carbide layer and the discontinuous zigzag shape of the transition layer, which fails to form a “pinning effect,” thereby weakening the interfacial bonding force of the composite material. In addition, when the sintering temperature is high, the cooling shrinkage rates of the copper matrix and diamond particles differ, which can easily lead to the formation of cracks at the interface. Therefore, further increasing the sintering temperature or pressure is not conducive to the interfacial bonding of the composite material and may even reduce the bending strength of the material.

From an industrial perspective, the vacuum hot-press sintering process offers several advantages, such as simple equipment requirements, low production costs, and the ability to achieve high-quality and dense composites. The process flexibility allows for precise control over the composite’s microstructure and properties, making it suitable for large-scale manufacturing [33]. Additionally, the cost-effectiveness of this method makes it particularly attractive for the consumer electronics market, where performance and price are critical factors.

The chromium–diamond/copper composite material holds significant promise for various high-performance applications due to its exceptional thermal conductivity and mechanical properties. One of the primary applications of chromium–diamond/copper composites is in the field of electronics, particularly for thermal management solutions. The high thermal conductivity of this composite material makes it an excellent candidate for heat sinks and thermal interface materials (TIMs) in electronic devices [34]. Effective thermal management is crucial for maintaining the performance and longevity of electronic components, especially in high-power applications, such as CPUs, and power electronics. In the aerospace and defense industries, materials with high thermal conductivity, low weight, and high mechanical strength are essential [35]. Chromium–diamond/copper composites can be used in various components, such as heat spreaders and thermal shields, where efficient heat dissipation is critical to ensure the reliability and safety of aerospace systems.

## 4. Conclusions

In this study, Cr–diamond/copper composite materials with Cr layer thicknesses of 150 nm and 200 nm were successfully prepared using vacuum hot-press sintering technology. The conclusions obtained from the experiment are as follows.

(1) Compared to the thermal conductivity of the diamond/copper composite materials without a Cr coating, the thermal conductivity of the composite material with a pre-coated Cr layer thickness of 150 nm increased by 266%, and the thermal conductivity of the composite material with a pre-coated Cr layer thickness of 200 nm increased by 242%, indicating that the introduction of the Cr layer effectively improved the thermal conductivity of the composite material.

(2) EDS analysis revealed the uniform distribution of Cr and C elements at the interface layer, confirming a reaction product with a thickness of approximately 650 nm.

(3) The thermal conductivity of the composites first increased and then decreased with rising sintering temperatures. At 1050 °C, the highest thermal conductivity of 593.67 W∙m^−1^∙K^−1^ was achieved. Further increases in sintering temperature or pressure had minimal impact on thermal conductivity.

(4) The added Cr layer reacts with diamond particles to form continuous, irregular carbides. These interfacial reactions create a “pinning effect,” strengthening the bond between the diamond particles and the copper matrix. This improved interfacial bonding enhances the composite material’s bending performance.

(5) Chromium-coated diamond/copper composite materials can be prepared through vacuum hot-press sintering at 1050 °C and 20 MPa, meeting high-power semiconductor component heat-dissipation requirements and providing industrial production references.

## Figures and Tables

**Figure 1:** Surface morphology of composite materials: (**a**) diamond/copper composite material; (**b**) Cr–diamond/copper composite material.

**Figure 2:** SEM images of diamond particles: (**a**) bare diamond particle (20 µm scale); (**b**) surface morphology of diamond particle (10 µm scale).

**Figure 3:** Interface morphology of Cr–diamond/copper composite materials: (**a**) interface; (**b**) interface amplification phase.

**Figure 4:** EDS schematic of diamond particles in the composites.

**Figure 5:** XRD schematic of diamond particles in the composites.

**Figure 6:** Interface scanning surface of Cr–diamond/copper composite materials: (**a**) interface scanning element distribution map; (**b**) interface line scanning element distribution curve.

**Figure 7:** Thermal conductivity of Cr–diamond/copper composite materials in the range of 298 K~573 K.

**Figure 8:** CTE curves of Cr–diamond/Cu composite materials.

**Figure 9:** The fracture morphology of composite materials prepared at a sintering temperature of 850 °C: (**a**) No.1 (diamond/copper composite material); (**b**) No.2 (Cr–diamond/copper composite material); (**c**) No.1 (1000×); (**d**) No.2 (1000×).

**Figure 10:** Fracture morphology of composite materials prepared at a sintering temperature of 1050 °C: (**a**) No. 3 (20 MPa); (**b**) No. 4 (25 MPa); (**c**) No. 3 (1000×); (**d**) No. 4 (1000×).

**Figure 11:** Fracture morphology of composite materials prepared at a sintering temperature of 1100 °C: (**a**) No. 5 (20 MPa); (**b**) No. 6 (25 MPa); (**c**) No. 5 (1000×); (**d**) No. 6 (1000×).

**Figure 12:** Surface morphology of diamond particles. (**a**) (100) face of the diamond (**b**) (111) face of the diamond.

**Table 1:** Thermal-performance-related parameters of Cr–diamond/copper composites.

No.	Chromium Layer Thickness/(nm)	Density /(g∙cm^3^)	Compactness /(%)	Thermal Diffusivity /(mm^2^∙s^−1^)	Specific Heat Capacity/(J∙g^−1^∙K^−1^)	TC /(W∙m^−1^∙K^−1^)
1	0	5.18	90.99	20.76	0.44	47.29
2	150	5.51	95.57	78.66	0.40	173.28
3	200	5.56	96.04	72.79	0.40	161.77

**Table 2:** Thermal diffusion coefficient, density, relative density, specific heat capacity, and thermal conductivity of Cr-plated diamond/Cu composite materials.

No.	Temperature /°C	Pressure /MPa	Density /(g∙cm^−3^)	Compactness /%	Thermal Diffusivity /(mm^2^∙s^−1^)	Specific Heat Capacity /(J∙g^−1^∙K^−1^)	TP /(W∙m^−1^∙K^−1^)
1 (without Cr)	850	20	5.27	92.5	63.40	0.38	127.14
2	850	20	5.40	94.6	199.87	0.39	417.52
3	1050	20	5.43	95.2	235.29	0.45	593.67
4	1050	25	5.58	97.8	251.55	0.40	590.14
5	1050	30	5.36	93.9	227.18	0.43	578.08
6	1100	20	5.40	94.6	265.68	0.41	580.54
7	1100	25	5.43	95.2	251.27	0.42	587.15

**Table 3:** Thermal diffusion coefficient of Cr-plated diamond/Cu composite material in the range of 298–573 K.

Sample	Thermal Diffusion Coefficient/(mm^2^∙s^−1^)			
	298 K	373 K	473 K	573 K
1050 °C, 20 MPa, 45 μm diamond	95.64±4.35	74.90±0.27	60.15±0.10	50.64±0.16
1100 °C, 20 MPa, 45 μm diamond	115.08±4.00	80.16±0.92	65.08±0.18	55.04±0.17
1050 °C, 20 MPa, 210 μm diamond	235.29±1.92	168.76±3.90	127.79±1.49	103.57±0.40
1050 °C, 25 MPa, 210 μm diamond	243.89±4.81	183.09±1.70	138.72±0.55	111.77±0.47
1100 °C, 20 MPa, 210 μm diamond	265.68±5.92	175.67±1.65	133.33±0.67	108.28±0.05
1100 °C, 25 MPa, 210 μm diamond	246.59±4.62	172.06±2.24	131.64±1.29	105.68±0.16

**Table 4:** Specific heat capacity of Cr–diamond/copper composite materials in the range of 298–573 K.

Sample	Specific Heat Capacity/(J∙g^−1^∙s^−1^)			
	298 K	373 K	473 K	573 K
1050 °C, 20 MPa, 45 μm diamond	0.38±0.01	0.39±0.00	0.49±0.00	0.56±0.00
1100 °C, 20 MPa, 45μm diamond	0.40±0.00	0.48±0.01	0.60±0.00	0.69±0.00
1050 °C, 20 MPa, 210μm diamond	0.45±0.01	0.60±0.02	0.75±0.01	0.86±0.01
1050 °C, 25 MPa, 210μm diamond	0.40±0.00	0.42±0.00	0.57±0.00	0.65±0.00
1100 °C, 20 MPa, 210μm diamond	0.41±0.01	0.47±0.00	0.61±0.00	0.71±0.00
1100 °C, 25 MPa, 210μm diamond	0.42±0.00	0.55±0.01	0.76±0.01	0.88±0.00

**Table 5:** Thermal expansion coefficient of Cr–diamond/Cu composite materials.

No.	Temperature /°C	Pressure /MPa	Thermal Expansion Coefficient /(×10^−6^K^−1)^		
			25~100 °C	25~200 °C	25~300 °C
1	1050	20	6.37	7.25	7.92
2	1050	25	6.48	7.31	7.99
3	1100	20	6.90	7.78	8.42
4	1100	25	6.73	7.69	8.38

## Data Availability

All data supporting the conclusions of this manuscript are included within the manuscript.
